RETRACTED

# microRNA-15b-5p encapsulated by M2 macrophage-derived extracellular vesicles promotes gastric cancer metastasis by targeting BRMS1 and suppressing DAPK1 transcription

**DOI:** 10.1186/s13046-022-02356-8

**Published:** 2022-04-22

**Authors:** Yi Cao, Yi Tu, Jianbo Xiong, Shengxing Tan, Lianghua Luo, Ahao Wu, Xufeng Shu, Zhigang Jie, Zhengrong Li

**Affiliations:** 1 Department of General Surgery, Jiangxi Province, The First Affiliated Hospital of Nanchang University, No. 17, Yongwai Zheng Road, Nanchang, 330006 People’s Republic of China; 2 Department of Pathology, The First Affiliated Hospital of Nanchang University, Nanchang, 330006 People’s Republic of China

**Keywords:** Gastric cancer, M2 macrophages, Extracellular vesicles, MicroRNA-15b-5p, BRMS1, DAPK1, Metastasis

## Abstract

**Background:**

Extracellular vesicles (EVs) derived from tumor-associated macrophages are implicated in the progression and metastasis of gastric cancer (GC) via the transfer of molecular cargo RNAs. We aimed to decipher the impact of microRNA (miR)-15b-5p transferred by M2 macrophage-derived EVs in the metastasis of GC.

**Methods:**

Expression of miR-15b-5p was assessed and the downstream genes of miR-15b-5p were analyzed. GC cells were subjected to gain- and loss-of function experiments for miR-15b-5p, BRMS1, and DAPK1. M2 macrophage-derived EVs were extracted, identified, and subjected to co-culture with GC cells and their biological behaviors were analyzed. A lung metastasis model in nude mice was established to determine the effects of miR-15b-5p on tumor metastasis in vivo.

**Results:**

miR-15b-5p was upregulated in GC tissues and cells as well as in M2 macrophage-derived EVs. miR-15b-5p promoted the proliferative and invasive potentials, and epithelial-mesenchymal transition (EMT) of GC cells. M2 macrophage-derived EVs could transfer miR-15b-5p into GC cells where it targeted BRMS1 by binding to its 3’UTR. BRMS1 was enriched in the DAPK1 promoter region and promoted its transcription, thereby arresting the proliferative and invasive potentials, and EMT of GC cells. In vivo experiments demonstrated that orthotopic implantation of miR-15b-5p overexpressing GC cells in nude mice displayed led to enhanced tumor metastasis by inhibiting the BRMS1/DAPK1 axis.

**Conclusions:**

Overall, miR-15b-5p delivered by M2 macrophage-derived EVs constitutes a molecular mechanism implicated in the metastasis of GC, and may thus be considered as a novel therapeutic target for its treatment.

**Supplementary Information:**

The online version contains supplementary material available at 10.1186/s13046-022-02356-8.

## Background

Gastrointestinal cancers reportedly account for 26% of the worldwide cancer burden and 35% of cancer deaths, and among these, gastric cancer (GC) has relatively higher prevalence in Asian populations [1]. Various kinds of risk factors have been discovered, including Helicobacter pylori infection, salt and fiber intake, obesity, smoking, age, and alcohol [2]. The major treatment modalities for GC include radical surgery, systemic therapy, and chemo or radiotherapy, but patients who succumb to metastatic tumors frequently present significant challenges for radical surgery and also tend to drug resistance [3]. Exploring the molecular mechanisms underlying metastasis of GC is essential for the developing efficient prevention and treatment modalities.

RETRACTED

Tumor-associated macrophages (TAMs) constitute critical players in the development of GC, and have been categorized into two major types, M1 and M2; although macrophage phenotype represents more of a continuum than a dichotomous state, and notably, M2 TAMs are potential therapeutic targets for GC treatment due to their immunosuppressive and pro-angiogenic phenotype [4]. Specifically, M2 macrophages have been reported to promote the metastatic potential of GC cells by secreting the chitinase 3-like protein 1 rotein in vivo [5]. In addition, M2 macrophages can release extracellular vesicles (EVs) to advance proliferative, migratory, and invasive potential of GC cells [6]. EVs [7] typically transfer their cargo of proteins, lipids, and RNAs from donor cells to recipient cells, thereby leading to changes in phenotypes within the tumor microenvironment [8]. miRNAs, which are a type of short noncoding RNAs, play essential roles in the pathological process of cancer by serving as oncomiRs or as tumor suppressors by means of numerous molecular mechanisms [9]. In particular, miR-15b-5p can promote the metastatic potential of GC cells by targeting PAQR3 [10]. The starBase database employed in the current study predicted binding sites between miR-15b-5p and BRMS1. The expression of the tumor suppressor gene BRMS1 is altered in different cancers, including GC, where its repression is noted to enhance invasion and metastasis of GC cells [11]. Further, the transcriptional activation of DAPK1 has been shown to be responsible for the metastasis-inhibiting effect of BRMS1 on hepatocellular carcinoma cells [12]. Notably, abnormal methylation of DAPK1 possesses positive correlation with the metastasis of GC [13]. Here, we aimed to evaluate the effect of miR-15b-5p in EVs from M2 macrophages on the metastasis of GC cells and specifically investigated putative molecular mechanisms involving the BRMS1/DAPK1 axis.

## Materials and methods

### Ethics statement

The Ethics Committee of The First Affiliated Hospital of Nanchang University approved the study protocol, which in accordance with the *Declaration of Helsinki*. All participants provided signed written informed consent. Animal experiments were undertaken following the approval of the Animal Ethics Committee of The First Affiliated Hospital of Nanchang University and were compliant with the Guide for the Care and Use of Laboratory animals published by the US National Institutes of Health.

RETRACTED

### Bioinformatics analysis

A GC-related miRNA expression dataset GSE97467 and a gene expression dataset GSE49051 were retrieved from the GEO database. Differential expression analysis was implemented to identify the differentially expressed miRNAs and genes using the R package "limma", with |logFC|> 1, *p* < 0.05 as the threshold. The starBase website was utilized to predict the targeting factors of miR-15b-5p.

### Sample collection

GC and adjacent normal tissues were surgically obtained from 49 patients diagnosed with GC at The First Affiliated Hospital of Nanchang University. Serum samples were obtained from these patients diagnosed with GC and from 20 healthy volunteers, and stored at -80 °C for later use. The patients with GC were followed up regularly for 5 years.

### Cell culture and treatment

The human monocyte macrophage line THP-1 was bought from the Cell Bank of Chinese Academy of Sciences (Shanghai, China), while HEK-293 T cells, GC cell lines (HGC-27, SNU-1, AGS and MKN-45), and the normal gastric epithelial cell line GES-1 were bought from Procell Life Science & Technology Co., Ltd. (Wuhan, Hubei, China). All cells were identified by short tandem repeat profiling. HEK-293 T cells, GC cell lines, and the normal gastric epithelial cell line were cultured in DMEM (Gibco, Grand Island, NY), comprising of 10% FBS, 100 U/mL penicillin and 100 μg/mL streptomycin. The THP-1 cell line was cultured in Roswell Park Memorial Institute (RPMI)-1640 medium (Gibco) containing 10% FBS, 100 U/mL penicillin and 100 μg/mL streptomycin. Plasmids of miR-15b-5p mimic, miR-15b-5p inhibitor and the corresponding NCs: mimic-NC and inhibitor-NC were designed by GenePharma Co., Ltd. (Shanghai, China).

pHAGE-puro plasmids and auxiliary plasmids pSPAX2 and pMD2 were co-transfected into 293 T cells with pSuper-retro-puro plasmids and auxiliary plasmids gag/pol and VSVG, cultured for 48 h, and the supernatant was collected. The supernatant was then subjected to centrifugation and filtration (0.45 μm filter) to collect virus. After 72 h, the supernatant was collected again for centrifugation and concentration. The two viruses were mixed and the concentration was determined. Lentiviral particles carrying overexpression (oe)-BRMS1, oe-DAPK1, and short hairpin RNA targeting BRMS1 (sh-BRMS1-1 and sh-BRMS1-2), sh-BRMS1 + DAPK1 or their separate NCs (Vector and sh-NC) were packaged into 293 T cells. The cells were trypsinized when they reached the exponential phase, and triturated into a cell suspension. Next, the suspension was seeded into 6-well plates (5 × 10^4^ cells/mL; 2 mL per well) for overnight culture at 37 °C. At 48 h after infection, the GFP expression efficiency was observed by using a fluorescence microscope (DMI4000B, Leica, Wetzlar, Germany).

RETRACTED

After 72 h of virus infection, the medium was substituted with a complete medium containing 2 mg/mL puromycin and the cells were further cultured for 5 days. shRNA sequences were designed by Life Technologies (https://rnaidesigner.thermofisher.com/rnaiexpress/sort.do) and synthesized by GenePharma. Detailed information is depicted in Supplementary Table 1.

### Induction and characterization of M2 macrophages

THP-1 cells were treated with 100 ng/mL 2-Acetoxy-1-methoxypropane (PMA; P8139, acquired from Sigma-Aldrich Chemical Company, St Louis, MO) for 24 h to induce differentiation into macrophages, and then with 20 ng/mL IL-4 (AF-200–04-5, Peprotech, Rocky Hill, NJ, USA) for 72 h to induce the differentiation into M2 macrophages. Cell surface antigens including CD11b, F4/80, CD206 and CD86, were tested by flow cytometry. Briefly, M2-polarized macrophages were trypsinized, rinsed with PBS, and resuspended in 100 μL PBS. Next, the cells were probed with antibodies against CD206-APC (550,889, BD Pharmingen, San Diego, CA, USA), CD86-V450 (560,357, BD Pharmingen), CD11b-PCy5.5 (740,861, BD Pharmingen) and F4/80-PE (565,410, BD Pharmingen) for 1 h. The cells were then resuspended with 0.5 mL PBS, filtered through a nylon mesh, and analyzed on a flow cytometer (Becton Dickinson, San Jose, USA).

### Fluorescence in situ hybridization (FISH)

The miR-15b-5p probe was customized by Exiqon (Woburn, MA, USA). Cells were soaked in 90%, 96%, 96%, 70%, and 70% ethanol for 5, 10, 5, 10 and 5 min, respectively. Next, the cells were washed with RNase-free PBS for 2–5 min, followed by incubation with proteinase K at 37 °C for 10 min and then with FISH working solution for 1 h. Following three standard sodium citrate (SSC) washes, the cells were probed with primary anti-CD206 antibody (ab64693, Abcam Inc., Cambridge, USA) for 2 h and re-probed with secondary antibody (ab150075, Abcam) for 90 min. Thereafter, DAPI (C1002, Beyotime Biotechnology Co., Shanghai, China) for nuclear staining was applied for 5 min. The cells were sealed with fluorescence decay resistant medium and five different fields were selected for observation under a FV-1000/ES confocal microscope. Double digoxin-labeled U6 (699,002–360, acquired from Exiqon) and Scramble-miR (699,004–360, acquired from Exiqon) probes were used as positive and negative controls, respectively.

RETRACTED

### Co-culture of M2 macrophages with Cy3-labeled GC cells

Cy3-labeled miR-15b-5p (miR-15b-5p-Cy3; GenePharma) was transfected into the AGS and MKN-45 cells using Lipofectamine 2000 reagents (11,668,019, Invitrogen Inc., Carlsbad, CA) to identify the delivery of miR-15b-5p in EVs. M2 macrophages expressing Cy3-miR-15b-5p were plated in 6-well plates and co-cultured with the AGS and MKN-45 cells in a Transwell chamber (3412, Corning Incorporated, Corning, NY, USA) for 2–4 days. Following three PBS rinses, AGS and MKN-45 cells were fixed, permeabilized, and stained with DAPI (C1002, Beyotime) followed by observation under a confocal microscope.

### Isolation and identification of EVs from M2 macrophages

M2 macrophages with good growth were cultured overnight in medium containing 10% serum without EVs. Upon 80—90% confluence, the supernatants from clinical serum samples and the cell culture medium were subjected to centrifugation (2000 g, 4 °C, 20 min) for the removal of cell debris. Next, the supernatants were gathered and centrifuged again (100,000 g, 4 °C) for a period of 1 h. Serum-free DMEM supplemented with 25 mM HEPES (pH = 7.4) was used for pellet suspension, and previously described high-speed centrifugation was undertaken again. The supernatant was then removed and the pellet was stored at -80 °C.

Observation of morphology of the isolated EVs was implemented under a TEM (JEOL USA Inc., Peabody, MA). DLS with a Zetasizer Nano ZS90 instrument (Malvern Instruments, Malvern, UK) was adopted to detect the size distribution of EVs at 532 nm. The expression of EV specific surface markers (TSG101 [ab125011, 1:1000], CD63 [ab134045, 1:1000], CD81 [ab109201, 1:5000], and Calnexin [ab22595]) was determined using Western blot analysis.

### Uptake of EVs by GC cells

The EVs isolated from M2 macrophages were labeled with PKH67 kit (KH67GL, Sigma-Aldrich). AGS and MKN-45 cells were cultured in the dish overnight, and then added with 10 μg PHK67-labeled EVs for 24 h of co-culture. The co-culture system was then soaked in 4% paraformaldehyde for 0.5 h, rinsed thrice with PBS, and permeabilized with 2% Triton X-100 for 15 min. Next, cells were blocked with 2% bovine serum albumin (BSA) for 45 min after three PBS washes. Thereafter, the cells were stained using DAPI (2 μg/mL) and mounted. Finally, fluorescence expression was detected using a fluorescence microscope.

### RNA isolation and quantitation

The total RNA was isolated from tissues with TRIzol reagents (16,096,020, Thermo Fisher Scientific Inc., Waltham, MA, USA). For the determination of mRNA, a reverse transcription kit (RR047A, Takara, Japan) was utilized. For miRNA, a polyA tailing detection kit (B532451, including universal PCR primers and U6 universal PCR primers; Sangon Biotechnology Co. Ltd., Shanghai, China) was selected. RT-qPCR was implemented by means of SYBR Premix Ex Taq™ (DRR081, TaKaRa) on an ABI 7500 instrument (Applied Biosystems, Foster City, CA, USA) or the TaqMan Gene Expression Assays protocol (Applied Biosystems). Primer sequences are illustrated in Supplementary Table 2. The expression of mRNA and miRNA was normalized to GAPDH and U6, respectively, while that of miRNA in EVs was normalized to synthetic caenorhabditis elegans (syn-cel)-miR-39. The fold changes were calculated by means of the 2^−ΔΔCt^ method.

RETRACTED

### Western blot analysis

Total protein was extracted, electrophoresed and then electroblotted to polyvinylidene fluoride membranes. Diluted primary antibodies: BRMS1 (ab134968, Abcam, Cambridge, UK), DAPK1 (ab200549, Abcam), E-cadherin (ab15148, Abcam), N-cadherin (ab18203, Abcam), Vimentin (ab137321, Abcam) and GAPDH (ab8245, Abcam) as well as secondary antibody goat anti-rabbit IgG (ab6721, 1: 5000, Abcam) or goat anti-mouse IgG (ab6789, Abcam) labeled by HRP were utilized. Image J software (National Institutes of Health, Bethesda, Maryland, USA) was utilized for band intensity quantification.

### ChIP assay

ChIP was implemented with the help of an EZ-Magna ChIP kit (EMD Millipore, Billerica, MA, USA) [14] using 1 μL BRMS1 rabbit antibody (ab134968, Abcam) and 1 μL IgG (as a NC, ab172730, Abcam) and the related primers were (Forward: 5’-CAGCGAGCGGGGTCTTAG-3’ and Reverse: 5’-GTAAAATGGCAACCCCAAAA-3’).

### Luciferase assay

Dual luciferase reporter gene plasmids containing the BRMS1 3’-UTR sequence (full length wild type [WT] and mutant type [MUT]) and DAPK1 promoter sequences (WT and MUT) were constructed. The reporter plasmids were subjected to co-transfection with miR-15b-5p mimic and mimic-NC plasmids into 293 T cells. The Dual-Luciferase® Reporter Assay System (E1910, Promega Corporation, Madison, WI, USA) was utilized to measure the luciferase activity.

### Transwell invasion assay

GC cells were plated into 24-well plates with 8 μm Transwell chambers (Corning) pre-coated with Matrigel. The detailed procedures were in light of the previous evidence [15]. The invading cells were counted and photographed using a laser confocal microscope (Olympus IX 71, Japan).

### Cell matrix adhesion test

The 96-well plate was coated with FN1/fibronectin (10 mg/mL, 10,838,039,001, Sigma-Aldrich) at 4 °C and then blocked with 1% BSA (A7030, Sigma-Aldrich). Cells were plated into the 96-well plate (5 × 10^4^ cells/well) and allowed to adhere at 37 °C for at least 10 min before three PBS washes. After a 2-week conventional culture, the cells underwent fixation in 4% paraformaldehyde for 30 min, staining with 0.5% crystal violet for 10 min, and treatment with 30% glacial acetic acid (A116172, Aladdin, China) for 15 min. After drying for 90 min, the cells were then imaged under a laser confocal microscope.

RETRACTED

### Establishment of lung metastasis models in nude mice

Healthy BALB/c nude mice (4–6 weeks old, acquired from Beijing Institute of Pharmacology of Basic Medical Sciences, Chinese Academy of Medical Sciences, Beijing, China) were raised in a SPF environment with 60—65% humidity at 22—25 °C under a 12-h light/dark cycle. The mice were given free access to food and water. The experiment began after one week of acclimation, and the health status of mice had been observed before the experiment. Stably infected GC cells were trypsinized into single cell suspension.

For the lung metastasis model, 5 × 10^5^ cells stably infected with lentiviruses carrying sh-NC + Vector, sh-BRMS1 + DAPK1, sh-NC + DAPK1, sh-BRMS1 + Vector, Vector and DAPK1 were injected into the mice via the tail vein. For the group treated with EVs, 20 μg of EVs was intraperitoneally injected into the mice every three days. A survival curve was plotted and analyzed.

### Hematoxylin–eosin (HE) staining

HE staining kit (C0105, Beyotime) was used for this assay. Briefly, the cells were dewaxed, rehydrated and washed. Subsequently, the cells were stained with hematoxylin staining solution for 5–10 min, then counterstained with eosin solution for 30 s—2 min, dehydrated with gradient alcohol (70%, 80%, 90% and 100%), cleared in xylene and sealed with neutral gum or other sealing agents before observation and photography under an inverted microscope (IX73, Olympus).

### Statistical analysis

Measured data were summarized as mean ± standard deviation. SPSS 21.0 software was utilized for data analysis. Significant differences were tested with the help of the unpaired *t*-test and one-way ANOVA with Tukey’s multiple comparisons test. The Kaplan–Meier method with log-rank test was selected for survival rate calculation. Correlation analysis was implemented using Pearson's correlation coefficient. A value of *P* less than 0.05 was considered statistically significant.

## Results

### miR-15b-5p transferred by M2 macrophage-derived EVs to GC cells facilitated the metastasis of GC cells

To address the relationship between EVs from M2 macrophages and miR-15b-5p, we first analyzed the GSE97467 dataset and found that miR-15b-5p was abundant in the EVs derived from M2 macrophages (Supplementary Fig. 1). RT-qPCR data was confirmatory, showing an increase in the expression of the miR-15b-5p in human GC tissues and GC cell lines (HGC-27, SNU-1, AGS and MKN-45) (Fig. 1A, B). RNA-FISH presented that the fluorescence signal of M2 marker CD206 and miR-15b-5p was enhanced in GC tissues with increased co-localization (Fig. 1C), indicating that the number of M2 macrophages and miR-15b-5p expression were increased in GC, and miR-15b-5p was expressed in M2 macrophages. As reflected by Ki67 staining, enhanced proliferation was observed in GC tissues (Fig. 1D). Then, we observed that the expression of E-cadherin was decreased, while levels of N-cadherin and Vimentin were enhanced in GC tissues (Fig. 1E).

RETRACTED

**Fig. 1:** Abundant expression of miR-15b-5p in M2 macrophage-derived EVs, GC tissues, and GC cell lines. **A** Expression of miR-15b-5p determined by RT-qPCR in adjacent normal and GC tissues from 49 patients with GC. **B** Expression of miR-15b-5p determined by RT-qPCR in GC cell lines HGC-27, SNU-1, AGS, and MKN-45, and normal gastric epithelial cell line GES-1. **C** Co-localization of CD206 and miR-15b-5p analyzed by RNA-FISH in GC tissues from 49 patients with GC (scale bar = 25 μm). **D** Ki67 staining of proliferation in GC tissues and adjacent normal tissues (scale bar = 50 μm). **E** Western blot analysis of E-cadherin, N-cadherin, and Vimentin protein expression in gastric cancer tissues and adjacent normal tissues. **F** Flow cytemetric analysis of CD11b, F4/80, CD206, and CD80. **G** Expression of M2 markers (Arg1, IL-10 and TGF-β) determined by RT-qPCR in M2 macrophages. **H** Morphological characterization of EVs observed under a TEM (scale bar = 100 nm). **I** Western blot analysis of EV surface makers (CD9, CD63 and TSG101) in the isolated EVs. **J** The size distribution of EVs analyzed by DLS. **K** Expression of miR-15b-5p determined by RT-qPCR in the EVs from M2 macrophages. **L** Expression of miR-15b-5p determined by RT-qPCR in the EVs from serum samples of 49 patients with GC and 20 healthy volunteers. **M** A curve showing the correlation of miR-15b-5p expression in EVs from serum samples of 49 patients with GC and the survival of patients. Each experiment was conducted three times independently. * p < 0.05, compared with adjacent normal tissues, GES-1 cell line, cell lysate or the EVs from undifferentiated M2 macrophages

Flow cytometric analysis suggested that the positive CD11b and F4/80 cells were over 90%, the expression of CD206 was positive while that of CD80 was negative in the differentiated M2 macrophages (Fig. 1F). At the same time, RT-qPCR results indicated an enhancement of the expression of M2 markers (Arg1, IL-10 and TGF-β) in the differentiated M2 macrophages (Fig. 1G). TEM showed that the EVs isolated from M2 macrophages were round or oval vesicles (Fig. 1H), and moreover, the size was in the range from 30 to 120 nm, analyzed by DLS (Fig. 1I). Further, the CD63, CD81, and TSG101 were positively expressed while Calnexin was not expressed in the isolated EVs (Fig. 1J). Therefore, EVs were successfully isolated from the M2 macrophages. RT-qPCR illustrated a higher expression of miR-15b-5p in the EVs from serum samples of patients with GC and from M2 macrophages (Fig. 1K, L). In addition, follow-up analysis revealed that the higher miR-15b-5p expression in EVs from serum samples of patients with GC was associated with worse prognosis (Fig. 1M).

RETRACTED

Next, we moved to investigating the effect of miR-15b-5p encapsulated by the EVs from M2 macrophages on GC. After 24 h of co-culture, AGS and MKN-45 cells could internalize the EVs (green fluorescence) secreted by M2 macrophages (Fig. 2A). Under a laser scanning confocal microscope, red fluorescence was observed in the pCDNA3.1-GFP-transfected AGS and MKN-45 cells following co-culture with the miR-15b-5p-Cy3-transfected M2 macrophages (Fig. 2B). RT-qPCR results depicted upregulated miR-15b-5p in the EVs from M2 macrophages transfected with miR-15b-5p mimic (EV-miR-15b-5p-mimic) (Fig. 2C). Following co-culture with the EVs, AGS and MKN-45 exhibited increased miR-15b-5p expression. Additionally, miR-15b-5p expression was also upregulated in AGS and MKN-45 cells treated with EV-miR-15b-5p-mimic (Fig. 2D). These results demonstrated that M2 macrophages could transfer miR-15b-5p to GC cells through EVs. Furthermore, colony formation and invasion of GC cells were enhanced in the presence of EV-mimic-NC, and a more prominent increase was noted in the presence of EV-miR-15b-5p-mimic (Fig. 2E, F). In addition, the extracellular matrix adhesion ability along with the expression of E-cadherin was decreased, while the expression of N-cadherin and Vimentin augmented in response to EV-mimic-NC. This trend was more pronounced in response to EV-miR-15b-5p-mimic (Fig. 2G, H, Supplementary Fig. 2A).

**Fig. 2:** miR-15b-5p transferred by M2 macrophage-derived EVs to GC cells where it promotes GC cell metastasis. **A** Uptake of M2 macrophage-derived EVs by AGS and MKN-45 cells observed under a fluorescence microscope (scale bar = 25 μm). **B** pCDNA3.1-GFP-transfected AGS and MKN-45 cells following co-culture with the miR-15b-5p-Cy3-transfected M2 macrophages observed under a confocal microscope (scale bar = 25 μm). **C** Expression of miR-15b-5p determined by RT-qPCR in M2 macrophages and the isolated EVs. **D** Expression of miR-15b-5p determined by RT-qPCR in AGS and MKN-45 cells treated with EV-mimic-NC or EV-miR-15b-5p-mimic. **E** Colony formation of GC cells in the presence of EV-mimic-NC or EV-miR-15b-5p-mimic. **F** Invasion of GC cells measured by Transwell assay in the presence of EV-mimic-NC or EV-miR-15b-5p-mimic. **G** Matrix adhesion ability of AGS and MKN-45 cells in the presence of EV-mimic-NC or EV-miR-15b-5p-mimic. **H** Western blot analysis of E-cadherin, N-cadherin, and Vimentin proteins in AGS and MKN-45 cells in the presence of EV-mimic-NC or EV-miR-15b-5p-mimic. Each experiment was conducted three times independently. * p < 0.05, compared with AGS and MKN-45 cells treated with mimic-NC, PBS, mimic-NC + Vector. #* p* < 0.05, compared with AGS and MKN-45 cells treated with EV-mimic-NC, miR-15b-5p mimic + Vector

RETRACTED

### miR-15b-5p targets BRMS1 in GC cells

To investigate potential downstream regulatory mechanisms of miR-15b-5p in GC, differential analysis of the GC-related GSE49051 dataset was applied, which revealed 2590 upregulated genes and 4165 downregulated genes in GC. BRMS1 was among the downregulated genes (Fig. 3A, B). Further GEPIA2 analysis showed an inverse correlation of BRMS1 expression with poor prognosis (Fig. 3C). For further verification, RT-qPCR was conducted, which confirmed reduced BRMS1 expression in GC tissues and cell lines (Fig. 3D, E).

**Fig. 3:** BRMS1 is a target of miR-15b-5p in GC cells. **A** A volcano plot of differentially expressed genes obtained from the GC-related GSE49051 dataset. **B** BRMS1 expression in the GSE49051 dataset. Red indicates GC samples and gray indicates normal samples. **C** Relationship between BRMS1 expression and survival of patients with GC, analyzed using the GEPIA2 database (http://gepia2.cancer-pku.cn/#index). **D** Expression of BRMS1 determined by RT-qPCR in GC tissues and adjacent normal tissues from 49 patients with GC. **E** Expression of BRMS1 determined by RT-qPCR in GC cell lines HGC-27, SNU-1, AGS and MKN-45, and normal gastric epithelial cell line GES-1. **F** Predicted miR-15b-5p binding sites in the 3’UTR of BRMS1 using the starBase database. **G** Binding of miR-15b-5p to BRMS1 confirmed by dual-luciferase reporter assay. **H** miR-15b-5p expression determined by RT-qPCR in AGS ad MKN-45 cells transfected with miR-15b-5p inhibitor. **I** Western blot analysis of BRMS1 protein in AGS and MKN-45 cells transfected with miR-15b-5p mimic or inhibitor. Each experiment was conducted three times independently. * p < 0.05, compared with adjacent normal tissues, GES-1 cell line, 293 T cells or AGS and MKN-45 cells transfected with mimic-NC. # *p* < 0.05, compared with AGS and MKN-45 cells transfected with inhibitor-NC

Then, the binding sites between miR-15b-5p and BRMS1 binding sites were predicted using the starBase database (Fig. 3F), which was further confirmed by a luciferase assay (Fig. 3G), indicating that miR-15b-5p could specifically target BRMS1. Moreover, miR-15b-5p expression was altered in GC cells. RT-qPCR results presented lower expression of miR-15b-5p in the presence of miR-15b-5p inhibition (Fig. 3H). Additionally, miR-15b-5p overexpression could downregulate the expression of BRMS1 whereas an opposite result was seen upon miR-15b-5p inhibition (Fig. 3I). These results suggested that miR-15b-5p targeted BRMS1 and inhibited its expression in GC cells.

RETRACTED

### miR-15b-5p potentiates the proliferation, invasion and EMT of GC cells by targeting BRSM1

To determine whether miR-15b-5p induces malignant phenotype of GC cells by targeting BRMS1, we first constructed plasmids overexpressing BRMS1 and verified the overexpression effect using RT-qPCR (Fig. 4A). Additionally, Western blot analysis illustrated a decline of BRMS1 following miR-15b-5p overexpression while further BRMS1 overexpression reversed this trend (Fig. 4B, Supplementary Fig. 2B). Moreover, miR-15b-5p overexpression potentiated the colony formation and invasion of GC cells while this effect was weakened by simultaneous overexpression of miR-15b-5p and BRMS1 (Fig. 4C, D). There was a downward trend in the extracellular matrix adhesion ability along with decreased E-cadherin expression yet increased N-cadherin and Vimentin expression in the presence of miR-15b-5p mimic + Vector. However, treatment with miR-15b-5p mimic + BRMS1 negated the aforementioned effects (Fig. 4B, E).

**Fig. 4:** miR-15b-5p facilitates the proliferation and invasion of GC cells by targeting BRSM1. **A** Expression of BRMS1 determined by RT-qPCR in AGS and MKN-45 cells overexpressing BRSM1. AGS and MKN-45 cells were transfected with miR-15b-5p mimic or combined with BRMS1. **B** Western blot analysis of BRMS1, E-cadherin, N-cadherin and Vimentin proteins in cells. **C** Colony formation of AGS and MKN-45 cells. **D** Invasion of AGS and MKN-45 cells measured by Transwell assay. **E** Matrix adhesion ability of AGS and MKN-45 cells. Each experiment was conducted three times independently. * p < 0.05, compared with AGS and MKN-45 cells transfected with Vector or mimic-NC + Vector. #* p* < 0.05, compared with AGS and MKN-45 cells transfected with miR-15b-5p mimic + Vector

### BRMS1 impedes metastasis of GC cells by upregulating DAPK1

We then focused on the downstream factors of BRMS1. The GSE49051 dataset was first analyzed, the results of which showed reduced expression of DAPK1 in GC samples (Fig. 5A). RT-qPCR data further confirmed the decline of DAPK1 expression in GC tissues and cell lines (Fig. 5B, C). The BRMS1 expression was positively correlated with the DAPK1 expression (Fig. 5D), suggesting that BRMS1 may regulate the expression of DAPK1 in GC cells. For further verification, we conducted relevant experiments in GC cell lines in vitro. As shown in Fig. 5E-G, BRMS1 was enriched in the -191 to -181 region of the DAPK1 promoter and promoted the transcriptional activation of DAPK1-WT rather than that of DAPK1-MUT. Additionally, treatment with sh-BRMS1-1 and sh-BRMS1-2 downregulated the protein expression of DAPK1 in AGS and MKN-45 cells, of which sh-BRMS1-1 showed superior silencing effects and was thus used for subsequent experiments. On the contrary, overexpression of BRMS1 promoted the protein expression of DAPK1 (Fig. 5H, I, Supplementary Fig. 2C).

RETRACTED

**Fig. 5:** BRMS1 positively correlated with DAPK1 in GC cells. **A** Expression of DAPK1 obtained from the GC-related GSE49051 dataset. Red indicates normal samples and gray indicates GC samples. **B** Expression of DAPK1 determined by RT-qPCR in adjacent normal and GC tissues from 49 patients with GC. **C** Expression of BRMS1 determined by RT-qPCR in GC cell lines HGC-27, SNU-1, AGS, and MKN-45, and normal gastric epithelial cell line GES-1. **D** Relationship between BRMS1 expression and DAPK1 expression analyzed by Pearson's correlation coefficient. **E** BRMS1 binding sites in the DAPK1 promoter region and mutation sequences of DAPK1. **F** Enrichment of BRMS1 in the DAPK1 promoter region in AGS and MKN-45 cells analyzed by ChIP. **G** BRMS1 binding to DAPK1 confirmed by dual-luciferase reporter assay in 293 T cells. **H** BRMS1 expression determined by RT-qPCR in AGS and MKN-45 cells treated with sh-BRMS1-1 and sh-BRMS1-2. **I** Western blot analysis of BRMS1 and DAPK1 proteins in AGS and MKN-45 cells sh-BRMS1 or BRMS1. Each experiment was conducted three times independently. * p < 0.05, compared with adjacent normal tissues, GES-1 cell line, IgG or AGS and MKN-45 cells treated with sh-NC. # *p* < 0.05, compared with 293 T cells or AGS and MKN-45 cells treated with Vector

Next, we constructed stably transfected AGS and MKN-45 cell lines with sh-NC + Vector, sh-BRMS1 + Vector, sh-BRMS1 + DAPK1 and sh-NC + DAPK1. As shown in Fig. 6A and Supplementary Fig. 2D, the expression of BRMS1 was decreased following treatment with sh-BRMS1 + Vector or sh-BRMS1 + DAPK1, while it was increased following treatment with sh-NC + DAPK1 or sh-BRMS1 + DAPK1, indicating the successful construction of stable cell lines. In addition, an upward trend in the colony formation and invasion of GC cells upon BRMS1 silencing was seen, which was reverted following DAPK1 overexpression or combined with BRMS1 silencing (Fig. 6B, C). Further, there was a downward trend in the extracellular matrix adhesion ability along with E-cadherin expression, while N-cadherin and Vimentin expression was augmented in the presence of BRMS1 silencing. Conversely, DAPK1 overexpression or combined with BRMS1 silencing resulted in a contrasting trend (Fig. 6A, D, Supplementary Fig. 2D).

RETRACTED

**Fig. 6:** BRMS1 represses the proliferation and invasion of GC cells via DAPK1 enhancement. AGS and MKN-45 cells were treated with sh-BRMS1, DAPK1, or both. **A** Western blot analysis of BRMS1, DAPK1, E-cadherin, N-cadherin, and Vimentin proteins in cells. **B** Colony formation of AGS and MKN-45 cells. **C** Invasion of AGS and MKN-45 cells measured by Transwell assay. **D** Matrix adhesion ability of AGS and MKN-45 cells. **E** HE staining analysis of the lung tissues of mice treated with sh-BRMS1, DAPK1, or both (scale bar = 50 μm). **F** Survival curve of nude mice treated with sh-BRMS1, DAPK1, or both. Each experiment was conducted three times independently. *n* = 8 for mice following each treatment. * p < 0.05, compared with AGS and MKN-45 cells or mice treated with sh-NC + Vector. #* p* < 0.05, compared with AGS and MKN-45 cells or mice treated with sh-BRMS1 + Vector

To further verify that BRMS1 can inhibit the metastasis of GC cells through DAPK1 in vivo, we established a lung metastasis model in nude mice. HE staining analysis showed that the lung metastasis was increased and the survival was shortened in mice treated with sh-BRMS1 + Vector, while the lung metastasis was decreased and survival was prolonged in the presence of sh-NC + DAPK1 or sh-BRMS1 + DAPK1 (Fig. 6E, F). Collectively, these data reflected that BRMS1 could impair the metastasis of GC cells by upregulating DAPK1.

### M2 macrophage-derived EVs facilitate the metastasis of GC by inhibiting DAPK1

Finally, to characterize whether miR-15b-5p delivered by M2 macrophage-derived EVs regulates the BRMS1/DAPK1 axis in GC, we co-cultured the EVs from M2 macrophages following different treatments with AGS and MKN-45 cells. To verify the effect of M2 macrophage-derived EVs containing miR-15b-5p on the metastasis of GC cells in vitro, Transwell experiments were applied, showing that the EV-miR-15b-5p mimic transfection promoted AGS and MKN-4 cell invasion compared with the EV-mimic-NC (Fig. 7A). It was found that the expression of BRMS1 and DAPK1 was decreased following treatment with EV-mimic-NC + Vector, and the trend was more obvious following treatment with EV-miR-15b-5p mimic + Vector. In contrast, the expression of BRMS1 and DAPK1 was increased upon treatment with EV-miR-15b-5p mimic + BRMS1 (Fig. 7B, Supplementary Fig. 2E).

RETRACTED

**Fig. 7:** M2 macrophage-derived EVs induce the metastasis of GC via DAPK1 impairment in vivo. **A** The invasion of AGS and MKN-4 cells treated with EV-miR-15b-5p mimic and EV-mimic-NC determined with Transwell assay (scale bar = 50 μm). **B** Western blot analysis of BRMS1 and DAPK1 proteins in cells treated with EV-mimic-NC + Vector, EV-miR-15b-5p mimic + Vector or EV-miR-15b-5p mimic + BRMS1. **C** Western blot analysis of BRMS1, DAPK1, E-cadherin, N-cadherin, and Vimentin proteins in cells treated with M2-EV + Vector and M2-EV + DAPK1. **D** Colony formation of AGS and MKN-45 cells treated with M2-EV + Vector and M2-EV + DAPK1. **E** Invasion of AGS and MKN-45 cells treated with M2-EV + Vector and M2-EV + DAPK1 measured by Transwell assay. **F** Matrix adhesion ability of AGS and MKN-45 cells treated with M2-EV + Vector and M2-EV + DAPK1. **G** HE staining analysis of the lung tissues of mice treated with M2-EV + Vector and M2-EV + DAPK1 (scale bar = 50 μm). **H** Survival curve of nude mice treated with M2-EV + Vector and M2-EV + DAPK1. Each experiment was conducted three times independently. *n* = 8 for mice following each treatment. * p < 0.05, compared with AGS and MKN-45 cells or mice treated with PBS + Vector. #* p* < 0.05, compared with AGS and MKN-45 cells treated with EV-mimic NC + Vector, or AGS and MKN-45 cells or mice treated with M2-EV + Vector. ^ *p* < 0.05, compared with AGS and MKN-45 cells treated with EV-miR-15b-5p mimic + Vector

To elucidate whether M2 macrophage-derived EVs promote the metastasis of GC by regulating the expression of DAPK1, we first transfected plasmids of Vector and DAPK1 into GC cells, which were then co-incubated with the M2 macrophage-derived EVs (M2-EV + Vector and M2-EV + DAPK1). As depicted in Fig. 7C and Supplementary Fig. 2F, the expression of DAPK1 was diminished in cells treated with M2-EV + Vector while an opposite trend was evident in cells treated with M2-EV + DAPK1. In addition, there was an enhancement in the colony formation and invasion of GC cells upon treatment with M2-EV + Vector whereas this trend was reverted following treatment with M2-EV + DAPK1 (Fig. 7D, E). Extracellular matrix adhesion ability was inhibited along with decreased E-cadherin expression but elevated N-cadherin and Vimentin expression, in the presence of M2-EV + Vector. Conversely, M2-EV + DAPK1 brought about a contrasting trend (Fig. 7C, F, Supplementary Fig. 2F). Furthermore, in vivo experiments with HE staining suggested that M2-EV + Vector promoted lung metastasis and shortened the survival in mice while a contrary result was noted in the presence of M2-EV + DAPK1 (Fig. 7G, H). Cumulatively, the findings demonstrated that M2 macrophage-derived EVs could accelerate the metastasis of GC by suppressing DAPK1*.*

RETRACTED

## Discussion

Increasing evidence has supported the potential application of EV-encapsulated miRNAs as novel biomarkers and therapeutic targets in GC [16, 17]. The findings unfolded a promoting effect of miR-15b-5p encapsulated by M2 macrophage-EVs on the metastasis of GC via disruption of the BRMS1/DAPK1 axis.

EVs from different cells present distinct miRNA profiles, which are critical cargoes in the molecular modulation of cancer and in reciprocal crosstalk among tumor cells, thus engaging in cancer progression [18]. miR-21 has been found to be directly transferred by exosomes from M2 macrophages into GC cells, where they enhance drug resistance and anti-apoptotic ability [19]. In addition, miR-130b-3p delivered by M2 macrophage-derived EVs is capable of stimulating the survival, migration, and angiogenesis of GC cells [6]. We discovered that M2 macrophage-derived EVs could encapsulate miR-15b-5p and transfer it to the recipient GC cells, where miR-15b-5p facilitated the metastatic properties of GC cells. Partially in agreement with these findings, miR-15b has been identified to be transferred from M2 macrophage-derived EVs into hepatocellular carcinoma cells where it promotes proliferative, migratory, and invasive properties of hepatocellular carcinoma cells [20]. In addition, en enhancement in miR-15b-5p was seen in GC tissues, cell lines, and plasma samples, and moreover, its overexpression stimulated GC metastatic properties [10], which was very much in accordance with the present results. Therefore, miR-15b-5p shuttled by M2 macrophage-derived EVs may be useful as a potential prognostic biomarker as well as a therapeutic target in patients with GC.

miRNAs have been well-established to interact with 3’UTR of specific target mRNAs and thus trigger the inhibition of their expression [21]. In the present investigation, miR-15b-5p was identified to bind to the 3’UTR of BRMS1 mRNA and adversely regulated its expression in GC cells. BRMS1 ceases metastatic properties of GC cells significantly by suppressing nuclear factor kappa-B signaling pathway activation [22]. These results suggested that the promoting effect of miR-15b-5p on the metastasis of GC cells was linked to its targeting of the BRSM1 gene and the resultant inhibition of BRSM1 expression.

Further analysis exhibited that BRMS1 could impede the metastasis of GC cells by upregulating the expression of DAPK1. Consistently, DAPK1 has been identified as a appealing transcriptional target of BRMS1 and the luciferase units of -200 to -80 bp region of the DAPK1 promoter can be enhanced by BRMS1 in hepatocellular carcinoma cells [12]. Enhanced DAPK1 expression induced by fentanyl, a drug commonly used for perioperative and postoperative analgesia, aids in the inhibition of the proliferative, invasive, and migratory potential of GC cells [23]. Additionally, methylation of the DAPK1 promoter correlates with the presence of nodal metastasis and advanced tumor stage [24]. Therefore, upregulated DAPK1 may be another essential mechanism for the metastasis suppressive action of BRMS1 in GC cells.

RETRACTED

Several miRNAs including miR-93 and miR-124-3p exhibit an inverse correlation with DAPK1 by which they can block the expression of DAPK1 through different mechanisms [25, 26]. In the current study, miR-15b-5p transferred by M2 macrophage-derived EVs demonstrated an inhibitory effect on the expression of DAPK1 through the mechanism of downregulating the BRMS1 expression. However, whether M2 macrophage-derived EVs could accelerate the metastasis of GC by suppressing DAPK1 in vivo in unclear and warrants verification in future research.

## Conclusion

Overall, our study indicated that M2 macrophage-EVs can transfer miR-15b-5p into GC cells and stimulate the metastasis of GC by downregulating the BRMS1/DAPK1 axis (Fig. 8). This newly identified mechanism can support a better understanding of the metastasis of GC, which can further aid knowledge for improving the clinical care of patients with GC. Although BRMS1 has been confirmed to be a target of many miRNAs, such as miR-125a and miR-93-5p [11, 27], due to the paucity of available evidence addressing the targeting between miR-15b-5p and BRMS1, further investigation is necessary. In addition, the effects of GC cells-derived EVs carrying miR-15b-5p on the microenvironment that can induce M2 type differentiation should be investigated in the future.

**Fig. 8:** Schematic diagram depicting the mechanism by which miR-15b-5p affects the metastasis of GC. EVs from M2 macrophages can transfer miR-15b-5p to GC cells where it is upregulated and targets BRMS1 to inhibit its expression. The expression of DAPK1 is thus suppressed and the metastasis of GC cells is ultimately accelerated

## Supplementary Information

**Additinal file 1: Supplementary Fig. 1.** The expression of miR-15b-5p in EVs derived from M2 macrophages in the GSE97467 dataset.

**Additional file 2: Supplementary Fig. 2.** A, Representative protein bands of figure 2H. B, Representative protein bands of figure 4B. C, Representative protein bands of figure 5I. D, Representative protein bands of figure 6A. E, Representative protein bands of figure 7B. F, Representative protein bands of figure 7C.

RETRACTED

**Additional file 3.**

## Data Availability

The datasets generated/analyzed in the current study are available.

## Abbreviations

EVs: Extracellular vesicles
GC: Gastric cancer
miR: MicroRNA
TAMs: Tumor-associated macrophages
CHI3L1: Chitinase 3-like protein 1
ncRNAs: Noncoding RNAs
PAQR3: Progestin and adipoQ receptor family member 3
BRMS1: Breast cancer metastasis suppressor 1
DAPK1: Death-associated protein kinase 1
GEO: Gene Expression Omnibus
NCs: Negative controls
oe: Overexpression
GFP: Green fluorescent protein
RT-qPCR: Reverse transcription quantitative polymerase chain reaction
SSC: Standard sodium citrate
DAPI: 4',6-Diamidino-2-phenylindole
TEM: Transmission electron microscope
DLS: Dynamic light scattering
